The article "Research Report on the Application of MEMS Sensors Based on Copper Oxide Nanofibers in the Braking of Autonomous Vehicles" was published in 2022. Journal: J Environ Public Health.

# Research Report on the Application of MEMS Sensors Based on Copper Oxide Nanofibers in the Braking of Autonomous Vehicles

**DOI:** 10.1155/2022/5852729

**Published:** 2022-09-05

**Authors:** Kuiyuan Guo, Xiaoqin Zhou

**Affiliations:** School of Mechanical and Aerospace Engineering, Jilin University, Changchun, Jilin 130025, China

## Abstract

Herein, we report a novel nanofiber as a humidity sensor applied to autonomous vehicles. We prepared copper oxide nanofibers by electrospinning, characterized the obtained materials by XRD, SEM, and TEM, and fabricated MEMS sensors based on copper oxide nanofibers. The humidity sensitivity performance of the sensor was tested in different humidity environments. We found that the MEMS humidity sensor based on copper oxide nanofibers can detect the change of humidity in the environment over a large humidity range. Its fast response/mixing speed (1 s), good stability, and sensitivity make it to fully adapt to the high speed of the car.

## 1. Introduction

As one of the basic substances that constitute life, water plays an inaccessible but important role in human production and life. In the environment of our daily life, water can be said to be innumerable, and it affects every bit of our lives all the time [1]. The term “humidity” usually refers to the amount of water vapor in the atmosphere. It is worth noting that humidity not only affects the comfort level of the human body but also interferes with the results of many experiments, which require us to detect and control the environmental humidity [2].

A humidity sensor is an important device used to detect environmental humidity, which is widely used in medical, biological, construction, and other fields [3]. The performance of the humidity sensor determines that only those materials with high sensitivity to humidity, rapid response, nontoxic, and nonpolluting materials are suitable for advanced humidity-sensitive materials [4]. At present, effective progress has been made in humidity sensors based on semiconductor metal oxides [5] and conductive polymers [6], and many different types of humidity sensors with good performance have been developed and put into practical applications. In addition, carbon-based materials have gradually become a hot spot for humidity sensors [7].

Among them, the humidity sensor based on semiconductor metal oxide has excellent sensitivity, can maintain good humidity sensitivity at room temperature, and can effectively detect humidity values in a wide humidity range, gradually becoming a research hotspot in the field of humidity sensing [8, 9]. For humidity sensors based on semiconductor metal oxides, the sensing mechanism is usually related to the change in the resistance of the humidity-sensitive material.

Copper oxide (CuO) is a typical p-type semiconductor metal oxide with a band gap of only 1.2 eV [10], which not only has high electrical conductivity but also has low production cost, easy preparation, nontoxic and harmless, and has gradually developed into a popular material in the field of humidity sensing [11]. According to research, the application of copper oxide can effectively reduce the cost of humidity sensing materials [12].

Copper oxide is a typical chemical resistance sensing material, and its sensing mechanism is inseparable from the change in the conductivity of the material itself caused by the adsorption of water molecules on the surface [13]. As shown in Figure 1, the adsorption of water molecules on the surface of copper oxide can be divided into physical adsorption and chemical adsorption [14]. Charge transfer is achieved by proton hopping between hydroxyl groups of the chemisorption layer [4]. The chemical adsorption layer of water molecules that has been formed will continue to accept water molecules and form a physical adsorption layer in the outer layer. According to the Grotthuss transport mechanism, a large number of water molecules are ionized to form hydronium ions, and the charge transfer is achieved by the hopping of hydrogen ions between adjacent water molecules [15]. This process will increase the electrical conductivity of the material, which will change the resistance of the copper oxide [16, 17]. It is because of the change of this resistance with humidity that the detection of the humidity value is realized.

It is worth mentioning that the operating temperature is always an important factor affecting the performance of the sensor [18, 19]. The operating temperature of the sensor will affect the electron mobility inside the material, thereby controlling the electrical conductivity of the material [20]. In the field of gas sensing, how to reduce the working temperature of the sensor is always a difficult problem because the working temperature is too high, which means the loss and waste of energy, which is in serious conflict with the current theme of energy conservation and emission reduction in the world [21, 22]. In addition, the high operating temperature will also affect the stability and sensitivity of the material, thereby reducing the service life of the sensor [12]. In contrast, the humidity sensor based on copper oxide shows relatively excellent humidity sensitivity even at room temperature, so no additional heating device is required, which not only reduces power consumption but also makes the sensor more portable [23–27]. There is no doubt that the humidity sensor based on copper oxide is more suitable for our living needs, whether from the perspective of cost and energy, or for convenience.

In addition to playing a huge role in medical, biological, and other fields, humidity sensors can also be applied to a new generation of automotive autonomous driving technology, as shown in Figure 2.

In this work, we fabricated a novel MEMS humidity sensor using copper oxide nanofibers for environmental humidity detection in autonomous vehicles. The material was synthesized by electrospinning technology. Our work aims to provide a guideline for mass production at an industrial level. The obtained sample was characterized by XRD/SEM and fabricated into a MEMS sensor. The MEMS sensor integrates a Pt wire for temperature measurement. We installed the sensor on the body behind the car tire. When the vehicle is running, the updraft rolled up by the tire will bring the water molecules on the ground to the sensor position, so as to feedback the humidity of the ground, and the sensor can be used for automatic driving braking.

## 2. Experiments

### 2.1. Materials and Methods

Ethanol (>99%) and copper chloride (CuCl_2_·6H_2_O) were purchased from Merck Company. Vinyl alcohol (PVA, Mw = 31,000–50,000) and vinylpyrrolidone (PVP, Mw = 1,300,000) were obtained from Sigma Aldrich. All chemicals were of analytical grade and were used as received without further purification.

We used electrospinning to prepare copper oxide nanofibers by electrospinning a mixture of copper chloride (CuCl_2_·6H_2_O) and polyvinyl alcohol (PVA). The specific method is to first dissolve the polyvinyl alcohol powder in deionized water, stir at 60°C for 5 h to obtain a 10 wt% PVA solution, and then add 20 wt% copper chloride solution and polyvinylpyrrolidone powder to the solution; after fully stirring for 12 h, inject the resulting solution into a 20 ml syringe equipped with a metal needle tip in a controlled electrospinning device. The applied voltage for electrospinning was 20 kV, the feeding rate of the mixed solution was 0.2 mL/h, and the distance between the glass substrate and the needle tip was 10 cm. Finally, the fibers obtained by electrospinning were peeled off with tweezers and placed in a crucible. The material was calcined at a temperature of 400 °C for two hours. Simultaneously remove organic components (PVP/PVA) in nanofibers.

### 2.2. Synthesis of CuO Nanofibers

The structure of the calcined CuO nanofibers was verified using the X-ray diffraction (XRD) technique (a Philips XRD diffractometer using Cu *Kα* (*Kα* = 1.540 Å and 2*θ* = 10–80 radiation as the X-ray source)). Scanning electron microscopy (SEM) images of calcined nanofibers were obtained using a LEO 1450 VP (Germany) instrument.

### 2.3. Humidity Sensitivity Test

The MEMS humidity sensor is fabricated by the following method. First, the sensing material and absolute ethanol are ground into a uniform paste, and the paste is applied on the surface of the central interdigitated electrode of the MEMS chip with a brush. The thickness of the sensing film is 100 *μ*m. After ethanol was volatilized, the device was aged at 250°C in ambient air to improve its stability and obtain a resistive MEMS humidity sensor.

In order to investigate the influence of gas concentration on the response, a gas distribution system (CGS-Beijing Ailite) is used to control the different humidity and then evaporated into the well-defined concentration of the target gas in the reaction chamber. We used dry air through pure water to control the humidity level inside the test chamber by adjusting the flow rates of dry air and humid air at room temperature. During these measurements, the humidity level in the room is also monitored by a standard hygrometer.

## 3. Results and Discussion

The schematic structure of the sensor is shown in Figure 3(a), in which the signal electrode is interdigitated, and the temperature electrode is Pt wire, which is formed by bending back and forth to form a temperature measuring electrode.  Figure 3(b) shows the MEMS humidity sensor behind the actual car tire. The sensor after the material is grown is shown in the illustration. When the car is running, the rotating tire rolls up the rising airflow, which will bring the moisture from the ground to the surface of the MEMS sensor. In this way, the humidity of the ground is detected in real time.

The X-ray diffraction pattern (calcined CuO nanofibers) of CuO nanofibers placed at 400°C for 2 h is shown in Figure 4. The CuO peaks appear at diffraction angles of 32/53°, 35/55°, 38/75°, 48/75°, 51/40°, 58/35°, 61/57°, 66/28°, 68/14°, 73/01°, and 75/28°, corresponding to reflection from (1 1 0), (0 0 2), (1 1 1), (−2 0 2), (0 2 0), (2 0 2), (−1 1 3), (−3 1 1), (2 2 0), (3 1 1), and (−2 2 2) planes, respectively. The strongest diffraction pattern viewed at 2*θ* = 35/55° suggests that CuO grows with a preferential orientation of (0 0 2) on the glass plate and illustrates the formation of the single-phase of monoclinic CuO. The resulting XRD spectrum is in good agreement with the 2*θ* values reported in JCPDS Card Nos. 48–1548.43.

Figures 5 and 6 are the SEM and TEM images of the obtained material after calcination at different magnifications. From the figures, we can observe that the calcined copper oxide nanostructures are slender and fibrous. This shows that we have successfully prepared copper oxide nanofibers that meet the experimental requirements by electrospinning.

Figure 7 shows the variation trend of the impedance of the MEMS humidity sensor with humidity in the range of 0–100% humidity. The experimental results show that under the low humidity level of 0–20%, the impedance of the sensor does not change significantly; it almost maintains the state of a horizontal line. In the humidity range of 20–100%, it can be observed that the impedance of the sensor decreases linearly with the increase of humidity, and the impedance drops from 230000 Ohm to 60000 Ohm. This shows that in the range of 20–100% humidity, the MEMS humidity sensor shows a good response state to the ambient humidity and has excellent potential for humidity measurement applications.

Then, in the humidity range of 0–100%, we detected the change in the impedance of the MEMS humidity sensor during the two changes of humidity rising and falling. The results are shown in Figure 8, where the red line represents the change of the sensor impedance under the humidity reduction condition and the black line represents the process of increasing humidity. From the figure, we can find that the impedance change of the sensor is very small, whether it is from low humidity to high humidity or the opposite process from high humidity to low humidity. This shows that the heat change generated when water molecules adsorb or desorb on the surface of the copper oxide nanofiber material has little effect on the output impedance of the sensor, further proving the excellent response and stability of the MEMS humidity sensor.

Figure 9 shows the response/recovery curve of the MEMS humidity sensor based on copper oxide nanofibers. From the figure, we can conclude that this type of sensor exhibits good reversibility during repeated experiments in the humidity range of 11–98%. It shows that the sensor has a very ideal ability for rapid response and recovery, and its response and recovery time is only about 1 s. Therefore, even in the process of high-speed driving, the sensor can timely and efficiently give feedback on the ground humidity.

Figure 10 shows the stability of the sensors in the one-month period. One can see that the resistance of the sensors changes slightly for different humidity cases, indicting the good humidity stability of the gas sensor.

Figure 11 shows the changing trend of the surface temperature and humidity of the sensor located behind the car tire during acceleration and deceleration while the car is driving. From the figure, we can find that when the car is accelerating, the surface temperature of the sensor increases, but its humidity decreases significantly. On the contrary, during the deceleration of the car, the temperature decreases and the humidity increases. This is because, in the same humidity environment, when the speed of the car increases, the rotational speed of the wheels also increases, which results in a stronger updraft, and the air rubs against the sensor surface to increase its temperature. However, the strong air movement causes fewer water molecules to be adsorbed on the sensor surface, which explains why the humidity decreases with increasing vehicle speed.

## 4. Conclusion

In this work, we prepared copper oxide nanofibers by electrospinning and fabricated MEMS sensors based on copper oxide nanofibers by traditional methods. The humidity sensitivity performance of the sensor was tested in different humidity environments. We found that the MEMS humidity sensor based on copper oxide nanofibers can detect the change of humidity in the environment over a large humidity range. Its fast response/mixing speed (1 s), good stability, and sensitivity make it to fully adapt to the high speed of the car. In addition, based on the significant changes in the humidity and temperature of the sensor during acceleration and deceleration, the MEMS sensor can also monitor the speed of the car, which can realize braking adjustment for autonomous driving.

## Figures and Tables

**Figure 1:** Schematic diagram of the humidity sensing mechanism of CuO.

**Figure 2:** The humidity sensor behind a car tire.

**Figure 3:** (a) The block diagram of the sensor. (b) MEMS sensor on a car, and the inset is a picture of the sensor growing material.

**Figure 4:** XRD of copper oxide nanofibers prepared by electrospinning.

**Figure 5:** SEM of copper oxide nanofibers at different magnifications.

**Figure 6:** TEM of copper oxide nanofibers at different magnifications.

**Figure 7:** The humidity sensing curve of a humidity sensor.

**Figure 8:** The hysteresis curve of the humidity sensor.

**Figure 9:** The humidity sensor response/recovery curve.

**Figure 10:** The stability of the sensors in the one-month period.

**Figure 11:** The changing trend of the sensor surface temperature and humidity during the acceleration/deceleration of the car.

## Data Availability

The data used to support the findings of this study are available from the corresponding author upon request.
